This article has been retracted.

# Presepsin Predicts Severity and Secondary Bacterial Infection in COVID-19 by Bioinformatics Analysis

**DOI:** 10.1155/2022/9914927

**Published:** 2022-09-06

**Authors:** Yufei Chang, Linan Liu, Hui Wang, Jinghe Liu, Yuwei Liu, Chunjing Du, Mingxi Hua, Xinzhe Liu, Jingyuan Liu, Ang Li

**Affiliations:** ^1^Department of Emergency, Beijing Ditan Hospital Capital Medical University, Beijing, China; ^2^Department of Critical Care Medicine Beijing Ditan Hospital, Capital Medical University, Beijing, China; ^3^Biomedical Innovation Center, Beijing Shijitan Hospital, Capital Medical University Beijing Key Laboratory of Emerging Infectious Diseases, China; ^4^Institute of Infectious Diseases, Beijing Ditan Hospital, Capital Medical University, China

## Abstract

**Introduction:**

Novel coronavirus pneumonia (COVID-19) is an acute respiratory disease caused by the novel coronavirus SARS-CoV-2. Severe and critical illness, especially secondary bacterial infection (SBI) cases, accounts for the vast majority of COVID-19-related deaths. However, the relevant biological indicators of COVID-19 and SBI are still unclear, which significantly limits the timely diagnosis and treatment.

**Methods:**

The differentially expressed genes (DEGs) between severe COVID-19 patients with SBI and without SBI were screened through the analysis of GSE168017 and GSE168018 datasets. By performing Gene Ontology (GO) enrichment analysis for significant DEGs, significant biological processes, cellular components, and molecular functions were selected. To understand the high-level functions and utilities of the biological system, the Kyoto Encyclopedia of Genes and Genomes (KEGG) pathway enrichment analysis was performed. By analyzing protein-protein interaction (PPI) and key subnetworks, the core DEGs were found.

**Results:**

85 DEGs were upregulated, and 436 DEGs were downregulated. The CD14 expression was significantly increased in the SBI group of severe COVID-19 patients (*P* < 0.01). The area under the curve (AUC) of CD14 in the SBI group in severe COVID-19 patients was 0.9429. The presepsin expression was significantly higher in moderate to severe COVID-19 patients (*P* < 0.05). Presepsin has a diagnostic value for moderate to severe COVID-19 with the AUC of 0.9732. The presepsin expression of COVID-19 patients in the nonsurvivors was significantly higher than that in the survivors (*P* < 0.05).

**Conclusion:**

Presepsin predicts severity and SBI in COVID-19 and may be associated with prognosis in COVID-19.

## 1. Introduction

Novel coronavirus pneumonia (COVID-19) is an acute respiratory disease caused by the novel coronavirus SARS-CoV-2, which is closely related to SARS-CoV [1, 2]. The virus is transmitted from person to person through close contact by both symptomatic and asymptomatic infected individuals through respiratory droplets and may also occur through aerosols or contact with pollutants [3]. COVID-19 was declared as a global pandemic on March 11, 2020 [4]. As of December 12, 2021, more than 268 million cases of COVID-19 have been reported worldwide including more than 5.2 million deaths, which seriously threatens the security of global public health [5].

Severe and critical illness, especially secondary bacterial infection (SBI) cases, accounts for the vast majority of COVID-19-related deaths [6]. Severe COVID-19 patients usually have low immunity and long hospitalization time. Meanwhile, most severe COVID-19 patients have undergone invasive operations such as tracheal intubation and are high-risk groups for secondary infection [7]. During this COVID-19 pandemic, SBI is one of the most common complications and an important cause of death in COVID-19 patients [8, 9]. However, the relevant biological indicators of COVID-19 and SBI are still unclear, which significantly limits the timely diagnosis and treatment.

Cluster of differentiation 14 (CD14) is a glycoprotein from the Toll-like receptor (TLR) family, which exists in two forms including mCD14 and sCD14 [10]. The formed complex through lipopolysaccharide-binding protein and lipopolysaccharide on bacterial surface could activate the expression of inflammation-related genes through signal transduction and promote the progress of inflammatory response [11]. Presepsin is an N-terminal fragment with a molecular weight of 13 kDa, formed by cleavage of sCD14 by protease D under inflammatory reaction [12]. Presepsin plays a role in recognizing different ligands of Gram-positive and Gram-negative bacteria and stimulating inflammatory responses [13]. Presepsin may be an effective and reliable biomarker for the identification of systemic inflammatory response syndrome caused by bacterial infection, especially Gram-negative bacteria [14]. However, the role of presepsin in COVID-19 has not been fully illuminated yet.

In this study, we screened out the DEGs in severe COVID-19 with and without SBI. By performing Gene Ontology (GO) enrichment analysis for significant differentially expressed genes (DEGs), significant biological processes, cellular components, and molecular functions were selected. To understand the high-level functions and utilities of the biological system, the Kyoto Encyclopedia of Genes and Genomes (KEGG) pathway enrichment analysis was performed. By analyzing protein-protein interaction (PPI) and key subnetworks, the core DEGs were found. As one of the key genes, the CD14 gene encoding presepsin may have the potential to be a marker of SBI in COVID-19.

## 2. Methods

### 2.1. Identification of DEGs

The keyword “Covid-19; Secondary bacterial infection” was entered in the GEO database, and the GSE168017 and GSE168018 datasets were selected and downloaded. GEO2R (http://www.ncbi.nlm. http://nih.gov/geo/geo2r/) was used to identify and extract up- or downregulated DEGs in the dataset. We set *P* < 0.01 and ∣fold change (FC) | >2 as screening criteria and used R to draw a volcano plot of DEGs.

### 2.2. Functional Analysis of DEGs

Functional analysis of DEGs was performed using the GO database. The signaling pathways of DEGs were investigated based on the KEGG. GO and KEGG analyses were performed using the Annotation Visualization and Integrated Discovery Database (DAVID, https://david.ncifcrf.gov/). We set *P* < 0.05 and false discovery rate (FDR) <5% as screening criteria, and plotted the graph with R.

### 2.3. Construction of PPI Network

The STRING database (http://string-db.org/) was used to construct a PPI network. We imported the gene list into STRING and used the default function to obtain the interaction relationship of protein.

### 2.4. Identification of Core Genes

The Cytoscape software was use for visualization. We used the MCODE plug-in in Cytoscape to find key subnetworks and then used the Cytohubba plug-in to analyze the core DEGs using the betweenness method.

### 2.5. Analysis of the Diagnostic Value

The GSE168017 dataset was used to analyze the expression of CD14. The receiver operating (ROC) curve was used to evaluate the diagnostic value of CD14, and the area under the curve (AUC) was calculated [15].

### 2.6. Presepsin and COVID-19

According to the literature (Table 1), the serum presepsin content of patients with mild and moderately severe COVID-19, as well as surviving and dead COVID-19 patients, was analyzed. The ROC curve was drawn to analyze the diagnostic value of presepsin content on the severity of COVID-19 patients.

### 2.7. Statistical Analysis

The data was described as mean ± standard deviation (SD). For statistical analysis, the two-sample *t*-test or one-way analysis of variance (ANOVA) were used. *P* value < 0.05 was regarded as statistically significant. GraphPad 8.0 (IBM company, USA) was used for statistical analysis.

## 3. Results

### 3.1. DEGs in Severe COVID-19 with and without SBI

The DEGs between severe COVID-19 patients with SBI and severe COVID-19 patients without SBI were screened through the analysis of GSE168017 and GSE168018 datasets. As shown in Figure 1, the volcano map was plotted. A total of 17716 genes were involved in the screening, and 521 genes were differentially expressed. Specifically, 85 DEGs were upregulated, and 436 DEGs were downregulated.

### 3.2. GO Enrichment Analysis

As shown in Figure 2, GO enrichment analysis was performed for significant DEGs. For biological process (Figure 2(a)), we selected 10 most significant processes including inorganic anion transport, potassium ion import across plasma membrane, response to parathyroid hormone, cellular monovalent inorganic anion homeostasis, cellular anion homeostasis, anion transmembrane transport, inhibitory synapse assembly, anion homeostasis, myeloid dendritic cell differentiation, and response to magnesium ion. For cellular component (Figure 2(b)), we selected 10 most significant components including synaptic membrane, Golgi lumen, collagen containing extracellular matrix, GABA-A receptor complex, GABA receptor complex, anchored component of membrane, post synaptic membrane, dendrite shaft, dendrite membrane, and chloride channel complex. For molecular function (Figure 2(c)), we selected 10 most significant function s including benzodiazepine receptor activity, GABA-gated chloride ion channel activity, inhibitory extracellular ligand-gated ion channel activity, bioactive lipid receptor activity, ligand-gated ion channel activity, ligand-gated channel activity, ligand-gated anion channel activity, GABA-A receptor activity, inorganic anion transmembrane transporter activity, and inward rectifier potassium channel activity. The results suggested the DEGs were associated with the ion transport, transmembrane, and related receptor activity.

### 3.3. KEGG Pathway Enrichment Analysis

To understand the high-level functions and utilities of the biological system, the KEGG pathway enrichment analysis was performed. As shown in Figure 3, 10 most significant pathways were screened out. GABAergic synapse, morphine addiction, neuroactive ligand-receptor interaction, retrograde endocannabinoid signaling, serotonergic synapse, nicotine addiction, GnRH secretion, axon guidance, taste transduction, PD-L1 expression, and PD-1 checkpoint pathway in cancer may be associated.

### 3.4. PPI Network Analysis

By analyzing PPI and key subnetworks, the core DEGs were found and indicated in red and orange (Figure 4). The specific top 15 core DEGs were shown in Table 2. Of note, the CD14 (with the score of 108) was screened out for further analysis. As one of the key genes, the CD14 gene encoding presepsin may have the potential to be a marker of SBI in COVID-19.

### 3.5. High Expression of CD14 mRNA in COVID-19 with SBI

As shown in Figure 5(a), the expression level of CD14 mRNA was significantly increased in the SBI group of severe COVID-19 patients (*P* < 0.01). Moreover, the diagnostic value of CD14 was studied. As shown in Figure 5(b), the AUC of CD14 in the SBI group in severe COVID-19 patients was 0.9429, indicating that CD14 has a certain clinical value in the diagnosis of SBI in severe COVID-19 patients.

### 3.6. High Expression of Presepsin in Severe COVID-19

Furthermore, the serum presepsin content of patients with mild, moderate, and severe COVID-19 was analyzed. As shown in Figure 6(a), the serum presepsin content of patients with moderate to severe COVID-19 was significantly higher than that of patients with mild COVID-19 (*P* < 0.05). As shown in Figure 6(b), the ROC analysis showed presepsin has a diagnostic value for moderate to severe COVID-19 with the AUC of 0.9732.

Finally, the presepsin levels in the survivors and nonsurvivors of COVID-19 patients were further analyzed. As shown in Figure 6(c), the serum presepsin content of COVID-19 patients in the death group was significantly higher than that in the survival group, suggesting that presepsin may be associated with prognosis in COVID-19.

## 4. Discussion

CD14 plays a key role in promoting innate immunity against Gram-negative bacteria by transferring LPS to MD-2/Toll-like receptor 4 (TLR4), [16]. The soluble form of the CD14 molecule (sCD14) can be used to predict bacterial infection in multiple infectious diseases [17]. Jose et al. reported sCD14 levels were significantly higher among COVID-19 patients independently of ICU admission requirement, indicating the role of sCD14 in COVID-19 immunopathology [18]. In our study, we also found that the expression level of CD14 mRNA was significantly increased in the SBI group of severe COVID-19 patients. Moreover, CD14 has a certain clinical value in the diagnosis of SBI in severe COVID-19 patients with the AUC of 0.9429.

Identifying the cause of infection for early and effective antimicrobial therapy is critical to minimize antimicrobial resistance and secondary infections, while monitoring serum procalcitonin (PCT) levels can help isolate bacteria. Infections are distinguished from viral infections and noninfectious inflammatory conditions [19]. Studies have shown that PCT and C-reactive protein (CRP) have very high sensitivity and specificity for the diagnosis of SBI, and PCT is better than CRP [20]. The diagnostic and prognostic ability of presepsin is comparable to that of PCT; however, it has an advantage over PCT. PCT is often elevated due to the secondary response of cytokines, resulting in an unsatisfactory early diagnosis of sepsis [21]. In addition, according to currently available methods, presepsin levels can be detected within 17 minutes, which is significantly shorter than the detection time of PCT [14]. But even so, most studies do not recommend the use of presepsin as a single biomarker for sepsis diagnosis, but in combination with other sepsis markers and traditional diagnostic tools such as bacterial culture [22]. Kaplan et al. reported the presepsin/albumin ratio (PAR) for screening sepsis patients requiring intensive therapy [23].

Presepsin as a soluble N-terminal fragment of the sCD14 subtype can be used to diagnose sepsis in patients with COVID-19 [18]. The serum presepsin content of patients with moderate to severe COVID-19 was significantly higher than that of patients with mild COVID-19 and has a diagnostic value for moderate to severe COVID-19. Importantly, the serum presepsin content of COVID-19 patients in the death group was significantly higher than that in the survival group, suggesting that presepsin may be associated with prognosis in COVID-19. At present, presepsin is mainly used for the diagnosis, stratification, and prediction of sepsis and its associated complications [24]. The most important feature of presepsin is that it increases significantly in the early stage of sepsis. Compared with other biomarkers such as PCT, the plasma presepsin concentration increases earlier, which can significantly distinguish sepsis from nonsepsis [14]. In addition, this early timing feature also endows presepsin the superior diagnostic ability, which can be used for early diagnosis of postoperative sepsis [25].

A prospective study of patients with sepsis indicated that presepsin could predict various complications of sepsis [26]. Other studies have also found that presepsin can be used as an independent predictor to distinguish whether ARDS is derived from or complicated by sepsis, thereby guiding the use of early antibiotics in sepsis before blood culture results are available [27]. Presepsin is not only associated with long-term mortality and overall survival but also has good diagnostic performance as an independent predictor in predicting mortality in hospitalized patients. It can be used as a supplementary factor for stratifying sepsis patients with different prognosis groups [26]. In addition, presepsin is effective in distinguishing between infected and noninfectious organ failure and helps clinicians determine patient prognosis [28].

Recently, more researchers focused on the application of presepsin in COVID-19. A retrospective study of a small sample of COVID-19 pointed out that presepsin increased immediately after CRP increased, so it is believed that presepsin can predict prognosis based on laboratory test results at admission, enabling clinicians to identify high-risk patients with COVID-19 and determine early stage treatment options [29]. A study with a sample size of 88 cases (including healthy controls) found that the expression level of presepsin gradually increased with the severity of the COVID-19, and there was a significant difference between different clinical types (*P* < 0.001) [30]. Another meta-analysis that pooled 6 cross-sectional studies included a total of 420 patients with COVID-19 found that presepsin could significantly distinguish severe/critical patients from other types of patients, with a weighted mean (WMD) cutoff value of 416.97 (95% CI: 125.03-708.90) ng/L [31]. Compared with other types of patients, the level of presepsin in severe/critically ill patients with COVID-19 will increase by 2.74 times, and the concentration of presepsin in dead patients is more than 3 times that in surviving patients (727 vs. 2,543 ng/L; *P* < 0.0001) [31]. The area under the ROC curve for predicting severe COVID-19 was 0.738 (95% CI: 0.684–0.786; *P* < 0.001), suggesting that presepsin assay can provide useful clinical information for predicting adverse outcomes of COVID-19 and guide clinical and treatment decisions [31]. However, there is still no consensus on the role of presepsin in COVID-19.

## 5. Conclusion

In this study, we screened out the DEGs in severe COVID-19 with and without SBI. By performing GO enrichment analysis for significant DEGs, significant biological processes, cellular components, and molecular functions were selected. To understand the high-level functions and utilities of the biological system, the KEGG pathway enrichment analysis was performed. By analyzing PPI and key subnetworks, the core DEGs were found. The CD14 expression was significantly increased in the SBI group of severe COVID-19 patients with the diagnostic value. The presepsin expression was significantly higher in moderate to severe COVID-19 patients with a diagnostic value. The presepsin expression of COVID-19 patients in the nonsurvivors was significantly higher than that in the survivors, suggesting that presepsin may be associated with prognosis in COVID-19. As one of the key genes, the CD14 gene encoding presepsin may have the potential to be a marker of SBI in COVID-19. However, the underlying mechanism remains to be studied, and clinical trials involving large sample sizes should be performed to further validate our results.

## Figures and Tables

**Figure 1:** Volcano plot of DEGs between groups with and without SBI in severe COVID-19 patients. Red indicates significantly upregulated genes in the SBI group, blue indicates significantly downregulated genes, and gray indicates genes with no significant difference. Criteria: ∣Log_2_ (fold change) | >2 and *P* value < 0.01.

**Figure 2:** GO enrichment analysis. (a) The biological processes, (b) cellular components, and (c) molecular functions enriched by DEGs.

**Figure 3:** KEGG pathway enrichment analysis. The biological pathways enriched by DEGs.

**Figure 4:** PPI network analysis. The core DEGs were indicated in red and orange.

**Figure 5:** CD14 expression and diagnostic value. (a) Serum CD14 expression levels in severe COVID-19 patients with and without SBI. (b) ROC curve analysis of the diagnostic value of CD14 for SBI in severe COVID-19 patients. ^∗∗^*P* < 0.01.

**Figure 6:** Presepsin expression and diagnostic value. (a) Presepsin levels in serum of patients with mild to moderate to severe COVID-19. (b) ROC curve of the diagnostic value of presepsin level on the severity of COVID-19 patients. (c) Expression levels of presepsin in serum of COVID-19 patients in survivors and nonsurvivors. ^∗^*P* < 0.05.

**Table 1:** Comprehensive literature list.

Year	Country	Literature
2022	South Korean	Predictive values of procalcitonin and presepsin for acute Kidney injury and 30-day hospital mortality in patients with COVID-19
2021	Egypt	Presepsin as a novel biomarker in predicting inhospital mortality in patients with COVID-19 pneumonia
2021	South Korea	Presepsin and monocyte distribution width as a useful early biomarker of severity in patients with COVID-19
Between October 2020 and July 2021	Pakistan	Diagnostic value of novel presepsin and inflammatory biomarkers in predicting the clinical course of COVID-19
2021	Turkey	The role of presepsin in predicting severe coronavirus disease 2019 pneumonia prognosis
2021	Japan	Simultaneous daily platelet count and presepsin measurement from the time of ICU admission may be useful for predicting inhospital mortality of patients with severe COVID-19
2020	Italy	A simple prognostic score based on troponin and presepsin for COVID-19 patients admitted to the emergency department: a single-center pilot study
2021	Japan	Serum stratifin and presepsin as candidate biomarkers for early detection of COVID-19 disease progression
2020	Japan	Presepsin as a predictive biomarker of severity in COVID-19: a case series

**Table 2:** Top 15 core DEGs.

Rank	Name	Score
1	TPH1	168
2	GAD2	161.2667
3	VIL1	108
3	CD14	108
5	GRM2	103.5333
6	HPCA	78
6	LGR5	78
6	HCRT	78
9	SLC12A5	46.43333
10	GABRA1	44.96667
11	KCNT1	26.7
12	KCNJ3	26.43333
13	IL17A	22
14	FGF23	14
14	SOST	14

## Data Availability

The datasets used and/or analyzed during the current study are available from the corresponding author upon reasonable request.
